# Optimization on Medical Material Distribution Management System Based on Artificial Intelligence Robot

This article has been retracted.

**DOI:** 10.1155/2021/5511299

**Published:** 2021-03-19

**Authors:** Ying Yang, Limin Dong, Hua Rong, Jing Wu

**Affiliations:** ^1^Department of Nursing, General Hospital of Taiyuan Iron & Steel Co.,Ltd., Taiyuan 030008, China; ^2^Department of Gynaecology and Obstetrics, General Hospital of Taiyuan Iron & Steel Co.,Ltd., Taiyuan 030003, China

## Abstract

The traditional medical material distribution management system method lacks systematic analysis and relies heavily on the subjective judgment of related operators, and it is easy to cause excessive or too little inventory, which leads to waste of operating costs. This study builds on a dedicated system for artificial intelligence robot logistics and aims to minimize the total cost of medical material ordering and distribution operations. In addition, in view of the constraints in the actual operation of the hospital, this study uses the concept of the spatiotemporal network to construct an ordering and distribution scheduling planning model of single material certainty, single material stochastic, and multiple material stochastic to help the hospital make optimal decisions and ensure the hospital's continuous and stable operation. In addition, after building the system, this study designs experiments to analyze the performance of this study system. The research shows that the model constructed in this paper has a certain effect and can provide a reference for the follow-up medical material distribution management system.

## 1. Introduction

At present, the ordering and distribution of medical supplies in domestic hospitals under general operating conditions mainly adopt contractual regular ordering and regular in-hospital delivery. First of all, hospital decision makers predict the total demand for medical supplies in the next year based on past historical data and rules of thumb, and then plan the most appropriate order cycle, order quantity, and minimum safety stock. Then, the hospital decision maker signs a procurement contract with the supplier. Finally, the supplier regularly distributes supplies to the hospital in accordance with the contract. The regular distribution within the hospital is also determined by a similar method. However, as far as the operating results of various hospitals are concerned, this method lacks a systematic analysis and is quite dependent on the subjective judgment of the relevant operators. Therefore, it is easy to cause too much or too little inventory, leading to waste of operating costs. In the past, the research on medical material management mainly focused on inventory and distribution management. However, these studies fail to express the changes in inventory and distribution of materials in different times and spaces and related restrictions and costs. Therefore, it is not complete at the analytical level. Based on this, taking the hospital as the standpoint, aiming at minimizing the total cost of medical supplies ordering and distribution operations, and aiming at the constraints in the actual operation of the hospital, *t,* this paper uses the concept of space-time network to separately construct a single material certainty, a single material randomness, and a variety of material random order and distribution scheduling planning models to help hospitals make optimal decisions and ensure the hospital's continuous and stable operation.

At present, the main problems faced by my country's medical institutions in the procurement of medical materials include a large number of suppliers available in the market, but most of them currently have an incomplete supplier evaluation index system. Most hospitals have changed the traditional procurement method of “ordering in large quantities and ordering in small batches” to the current procurement method of “ordering in multiple batches and ordering in small quantities.” Under the premise of maintaining a certain inventory, the hospital minimizes the inventory and implements zero inventory management of medical materials, thereby reducing logistics costs and improving capital utilization. However, it is difficult to respond quickly to urgently needed medical supplies. That is, no corresponding procurement plans have been made for different medical supplies. In terms of internal distribution and transportation of medical supplies, domestic medical institutions generally arrange for relevant personnel to carry out special management. Moreover, it is necessary to record from the entry of the department staff who need to receive medical supplies to the registration of receipt and inventory inspection, and the medical supplies are transported by the internal delivery personnel with the help of handling tools. Under normal circumstances, there is a positive relationship between circulation and handling costs, inventory, and turnover. At present, in the internal circulation of medical supplies, the main problem is that the degree of information management of the materials used is low, and the material distribution personnel pick up the goods manually and use simple carts and other tools to receive medical materials. This is inefficient and unsafe, which invisibly increases logistics management costs.

For a long time, domestic hospital institutions have had problems with indiscriminate medicine and chaotic medicine supply systems. The hospital pharmacy matches the bonus sales function, which makes the selling price of drugs with lower actual costs become artificially high. Many pilot hospitals said that after the implementation of the “Zero Drug Plus” policy, due to the ambiguity of the original medical system property rights, all levels of hospitals were not very enthusiastic about reforms, which led to large “policy losses” in various hospitals. At this time, pharmacy trusteeship emerged as a way to reduce hospital losses [1]. Pharmaceutical companies not only have to pay custody fees to the hospital, pay the salaries of staff such as pharmacy warehouses, but also bear the pressure of personnel management and drug inventory management. Moreover, the hospital does not need to consider the management and operation issues brought about by the original pharmacy and instead focuses more on medical services, which is conducive to enhancing the competitiveness of the hospital [2]. In addition, for pharmaceutical companies, reducing intermediate links, lowering public relations fees, saving logistics costs, and achieving economies of scale have become the main ways to achieve profits [3]. Therefore, for the overall logistics planning of medical material ordering and distribution, it is worthwhile to study the practical application value and academic reference value to effectively control the cost of the entire drug supply chain while meeting the patient's drug needs.

## 2. Related Work

The literature [4] proposed an economic order quantity (EOQ) model with time-varying demand and purchase price to analyze the impact of the development of spoiled items on inventory management. On the basis of in-depth analysis of production materials and demand probability distribution of combat-ready medical materials, by increasing and adjusting the constraints and assumptions of demand data probability distribution, delivery time, and out-of-stock costs, the literature [5], on the basis of the classic EOQ inventory model, established three optimized EOQ inventory models with multiple factors such as quantitative inventory and uncertain inventory, known parameters, and random variables. The literature [6] proposed an E00 model in which both demand and purchase price are time-varying, proving that the model's total inventory cost objective function is a convex function under given conditions. Moreover, the literature gives an algorithm for seeking the best purchase times and service levels and performs numerical simulation and sensitivity analysis on the model.

In the background of multidrug ordering problems in hospitals, based on the theory of metamorphic inventory, the literature [7] established a mathematical model with inventory space as the constraint condition under the premise of allowing out-of-stock and having lead time and verified the validity of the model through numerical examples. The literature [8] proposed an optimized medical equipment ordering strategy and gave several formulas to determine the most reasonable order form. The literature [9] combines Six Sigma management and lean production methods to improve the hospital's inventory management of important medical equipment. The literature [10] constructed a VMI model for a single supplier and multiretailer supply chain.

## 3. Model Building

In actual operation, in order to allow the planned medical materials ordering and distribution operations to be stably executed, the relevant operators will regularly check whether the set standards of the medical material procurement system (such as the order quantity of various medical materials, minimum safety inventory, and other parameters) meet the actual needs, and replan the subsequent remaining operations according to the new medical material demand information to maintain the safe supply of materials [11]. This thesis uses the “Dynamic Decision Framework” for planning and scheduling on the time axis of the deterministic medical material ordering and distribution planning scheduling model and divides the time axis into two parts. Among them, one part is the “decision-making stage” that is closer to the point of use of medical materials [12]. The other part is to remove the decision-making period, and the period farther away from the time point of material use is called the “reference period.” In response to the needs of hospital departments, medical material assignment operations are carried out, and the new medical material demand information that is obtained every other fixed period (equal to the decision period) is again reassigned to the medical material ordering and distribution planning scheduling mode until the end of the planning period to obtain the results of medical material ordering and delivery scheduling that more closely met the actual needs [13]. In addition, the scheduling results during the decision-making period can be regarded as the determined medical material assignment operation range, and the scheduling results outside the decision-making period can provide reference values for the execution of this decision. After this reference value is compared with the scheduling results in the next stage's decision period, the degree of change in two different periods can be obtained [14]. This study builds on a dedicated system for artificial intelligence robot logistics.

The parameters of the model constructed in this study are shown in Table 1.

Based on the above description, the deterministic planning model can be expressed as follows:

(1) $$\begin{array}{c} \text{Min }Z=\sum_{ij\in SW}\left(px_{ij}+c\right)\delta_{ij}+\sum_{ij\in }dx_{ij}+\sum_{ij\in HA}\left(h_{w}+h_{d}\right)x_{ij}, \end{array}$$

(2) $$\begin{array}{c} \sum_{j\in NM}x_{ij}\delta_{ij}-\sum_{k\in NM}x_{ki}\delta_{kj}=a_{i},\;\forall i\in NM, \end{array}$$

(3) $$\begin{array}{c} l_{ij}\leq x_{ij}\leq u_{ij},\;\forall_{ij}\in AM, \end{array}$$

(4) $$\begin{array}{c} x_{ij}\in I,\;\forall_{ij}\in AM, \end{array}$$

(5) $$\begin{array}{c} \delta_{ij}=0\text{ or }1,\;\forall_{ij}\in AM. \end{array}$$

The objective formula (1) is the formula for minimizing the total cost of medical supplies ordering and distribution operations, which includes the purchase cost of supplies, in-hospital distribution costs, and inventory retention costs [15]. Constraint (2) is the conservation constraint of node flow [16]. Constraint condition (3) is the upper and lower limit of the flow rate of each node [17]. Constraint (4) is the integer limit of the node line flow [18]. Constraint (5) is the 0–1 limit of the 0–1 variable [19].

This paper designs an effective heuristic algorithm for this deterministic programming model [20]. The specific steps of this solution are as follows (Figure 1):

- Step 1: initialize the parameters. The algorithm parameters are set, including the number of simulated rounds *M*, the number of deterministic demand events N, and the model data is input, including the maximum safety stock of the hospital warehouse/department, safety stock, and initial stock, various cost data, and other relevant parameter data.
- (ii)Step 2: we set *m* = *l*. *m* is the number of simulation rounds.
- (iii)Step 3: the demand for medical supplies for each department at various points in time is generated, and this demand is substituted into the deterministic scheduling model.
- (iv)Step 4: with the goal of minimizing the total cost of the medical system during the planning period, the results of the hospital's medical material ordering and distribution throughout the planning period are solved. The scheduling results in the decision-making period are used as the determination results to carry out the distribution of medical supplies during the decision-making period. Moreover, the scheduling results of the previous decision period can be used as input data for the current decision period.
- (v)Step 5: the medical material demand of each department in the remaining planning period is continued to be generated, and the remaining total order cost of the medical system in the remaining planning period is taken as the goal to solve and obtain the remaining ordering and distribution scheduling results.
- (vi)Step 6: steps 4 and 5 are repeated until the ordering and distribution schedules for the entire planning period are all determined. Determine whether the conditions are met? If yes, proceed to the next step: otherwise, *m* = *m* + *l*, and return to step 4.
- (vii)Step 7: the optimal planning results and total operating costs are recorded. In operation, the two mathematical planning software programs MATLAB and CPLEX are combined in this thesis, and the arithmetic program is written in the MATLAB environment, and the mixed integer linear programming function cplexmilp () of CPLEX is called to solve. The specific calculation process of the algorithm is shown in Figure 1.

In order to facilitate the construction of the model and define the limitations of the use of the model, this paper proposes the basic assumptions of the following model [21] and Table 2.

1. The hospital is regarded as a standpoint and minimizing the total cost of medical supplies ordering and in-hospital distribution is taken as the goal.
2. The potential demand for medical supplies at each time node is random and conforms to a normal distribution.
3. The planning period for medical supplies ordering and distribution is one year (52 weeks), and the ordering of supplies and in-hospital supplies delivery is once a week.
4. The maximum storage capacity and safety stock of hospital warehouses and departments are known and fixed.
5. The hospital warehouse and various departments have a certain amount of inventory in the early stage of planning.
6. The maximum weekly output of the supplier is known and fixed.

Based on the above description, the stochastic programming model can be expressed as follows:

(6) $$\begin{array}{c} \text{Min }f, \end{array}$$

(7) $$\begin{array}{c} \mathrm{Pr}\left\{\sum_{ij\in SW}\left(px_{ij}+c\right)\delta_{ij}+\sum_{ij\in WD}dx_{ij}+\sum_{Ij\in HA}\left(hw+hd\right)x_{ij}+\sum_{i\in D}y_{i}t\leq \bar{f}\right\}\geq \alpha , \end{array}$$

(8) $$\begin{array}{c} \mathrm{Pr}\left\{\sum_{ij\in SW}xi_{j}\delta_{ij}-\sum_{k\in NM}x_{ki}\delta_{kj}=a_{i}\right\}\geq \beta ,\;\forall i\in NM, \end{array}$$

(9) $$\begin{array}{c} \mathrm{Pr}\left\{l_{ij}\leq x_{ij}\right\}\geq \lambda ,\;\forall_{ij}\in HA, \end{array}$$

(10) $$\begin{array}{c} x_{ij}\leq u_{ij},\;\forall_{ij}\in HA, \end{array}$$

(11) $$\begin{array}{c} l_{ij}\leq x_{ij}\leq u_{ij},\;\forall_{ij}\in RM, \end{array}$$

(12) $$\begin{array}{c} x_{ij},y_{ij}\in I,\;\forall_{ij}\in AM, \end{array}$$

(13) $$\begin{array}{c} \delta_{ij}=0,1,\;\forall_{ij}\in AM. \end{array}$$

The objective function (6) is to minimize the total cost of medical material ordering and distribution under random demand, and its specific components are reflected in formula (7): the first item in the total cost is the ordering cost of medical supplies, the second item is the internal distribution cost of the hospital, the third item is the inventory detention cost of medical supplies in the warehouse and the department, and the fourth item is the out-of-stock cost due to the inability to meet the needs of the departments. Equation (7) indicates that the target value of the model is the minimum value taken by the target function at the confidence level. Constraint (8) indicates that all nodes satisfy the conservation of traffic when the confidence level is ||. The constraint (9) indicates that the inventory of warehouses and departments must be higher than the safety stock when the confidence level is five. The constraints (10) and (11) are the upper and lower flow constraints of other pitch lines. The constraints (12) and (13) are the integer limit and O-1 limit of each decision variable.

The multilayered space-time network structure for medical material ordering and distribution was constructed. Each layer of the network represents a medical material so that the spatial and temporal distribution of different medical materials is distinguished. Elements such as nodes and node lines included in the space-time network have been described in detail in the foregoing. The symbol description is shown in Table 3 [22].

(14) $$\begin{array}{c} \text{Min }\bar{f}, \end{array}$$

(15) $$\begin{array}{c} \mathrm{Pr}\left\{\sum_{m\in N}\left(\sum_{ij\in SW}\left(p^{n}x_{ij}^{n}+c^{n}\delta_{ij}^{n}\right)+\sum_{ij\in WD}d^{n}x_{ij}^{n}+\sum_{Ij\in HA}\left(h_{w}^{n}+h_{d}^{n}\right)x_{ij}^{n}+\sum_{i\in D}y_{i}^{n}t^{n}\right)\leq \bar{f}\right\}\geq \alpha , \end{array}$$

(16) $$\begin{array}{c} \mathrm{Pr}\left\{\sum_{ij\in SW}x_{ij}^{n}-\sum_{k\in NM}x_{ki}^{n}=a_{i}^{n}\right\}\geq \beta ,\;\forall i\in NM,\forall n\in N, \end{array}$$

(17) $$\begin{array}{c} \mathrm{Pr}\left\{l_{ij}^{n}\leq x_{ij}^{n}\right\}\geq \lambda ,\forall_{ij}\in HA^{n},\;\forall_{ij}\in HA^{n},\forall_{n}\in N, \end{array}$$

(18) $$\begin{array}{c} \sum_{m\in N}x_{ij}^{n}\leq um_{ij},\;\forall_{ij}\in HA^{n},\forall_{n}\in N, \end{array}$$

(19) $$\begin{array}{c} x_{ij}^{n}\leq \delta_{ij}^{n}u_{ij}^{n},\;\forall_{ij}\in SM^{n},\forall_{n}\in N, \end{array}$$

(20) $$\begin{array}{c} l_{ij}^{n}\leq x_{ij}^{n}\leq u_{ij}^{n},\;\forall_{ij}\in RM^{n},\forall_{n}\in N, \end{array}$$

(21) $$\begin{array}{c} x_{ij}^{n},y_{ij}^{n}\in N,\;\forall_{ij}\in AM^{n},\forall_{n}\in N \end{array}$$

(22) $$\begin{array}{c} \delta_{ij}^{n}=0,1,\;\forall_{ij}\in AM^{n},\forall_{n}\in N. \end{array}$$

The objective function (14) is to minimize the total cost of medical material ordering and distribution under random demand, and its specific components are reflected in formula (15): the first item of the total cost is the ordering cost of medical supplies, the second item is the internal distribution cost of the hospital, the third item is the inventory retention cost of medical supplies in warehouses and departments, and the fourth item is the cost of out-of-stock due to random demand. Equation (15) indicates that the target value of the model is the target function to obtain the target value, and the confidence level is a*α*. Formula (16) indicates that the confidence level that all nodes satisfy the conservation of flow is *β*. Equation (17) indicates that the inventory of warehouses and departments is higher than the confidence level of safety stock. Formula (18) indicates that the total amount of various materials stored in warehouses and departments cannot exceed the maximum inventory capacity. Formula (19) is used to judge whether the hospital orders. Formula (20) is the upper and lower limit flow restrictions of other node lines. Formulas (21) and (22) are the nonnegative integer limit and 0–1 limit of each decision variable.

## 4. Real-Time Data Collection and Management System

Since the development of hospital informatization in the 1980s, the application level of hospital information has been rapidly improved. From the initial stand-alone manual management to the hospital's local system network, to the later construction of hospital information integration and the establishment of regional disease control centers, it shows that we have made great progress. In the early stages of development, due to limitations in technology, capital, and staffing, it is quite difficult to realize real-time monitoring of hospital information and scientific and effective management. However, with the continuous development of bioinformatics, predictive and early warning technology, and wireless networks, how to make full use of information technology to accurately monitor influenza in real time and to realize the prediction and early warning of influenza virus and the reasonable distribution of medical supplies on the basis of monitoring has become the focus of real-time influenza monitoring information. The influenza real-time data collection and management system is built to realize the informatization and intelligence of regional influenza prevention and control. Based on the analysis of the existing influenza center system, the system takes various types of influenza monitoring data (including disease changes, patient data in and out of hospital, and epidemiological data) as the core and uses the spread map analysis on the geographic information system as an indicator to collect, process, analyze and research influenza data in real time to create a unified, stable, and efficient, comprehensive forecast and early warning system to realize the monitoring and early warning of the influenza epidemic. The system is the information flow channel of the regional decision support system. It realizes the real-time collection of influenza information and the unified report of the epidemic situation and illness report. That is, it reflects the dynamic situation of the influenza epidemic every day, dynamically reflects the distribution of influenza patients in various hospitals, and comprehensively reflects the conditions of influenza patients.

By using the same coding principles, this paper develops a hospital information system that can realize information intercommunication and sharing and establishes a real-time data collection and management system for influenza that covers the entire region through the reasonable allocation of resources.  Figure 2 shows the system technical architecture diagram, which mainly includes data sources, data platforms, database management, data analysis modules, application management layers, and access layers. The data source is mainly connected with disease information systems of disease control centers, hospitals, and communities at all levels, which uniformly report relevant influenza data. The acquired data is collected and exchanged through the data warehouse platform. First, extract and verify the collected real-time data. Then, the subject database is integrated, reconstructed, stored, and managed by category. The stored data includes current and historical data. Finally, the data analysis module displays the analysis results in various views. The application service layer provides all information application services, and relevant data is extracted according to different needs.

Figure 3 analyzes the basic functions of the flu real-time data collection and management system from the perspective of the overall function of the system. It mainly includes five modules: regional distribution of influenza, patient information management, medical supplies management, data management, and remote consultation management.

1. Regional distribution of influenza: through the information sharing of the hospital information system of each hospital, the distribution map of the patients in each hospital, the distribution number of suspected cases, the latest geographical information map of the temporal and spatial distribution of influenza, and relevant real-time epidemic information can be displayed.
2. Patient information management: the system can store the personal information of infected patients, including name, age, gender, hospital, home address, and contact information. Moreover, it can also manage patient track information to determine areas that may cause high infection rates. In addition, it can also store patient information to provide data support for subsequent medical research.
3. Medical supplies management: it manages the basic information of related hospitals, including the location of the hospital, the level of the hospital, the diagnosis and treatment technology, the number of medical staff, and the number of patients admitted. Moreover, it manages the use of influenza-related medical supplies, the amount of ordering, and the amount of distribution.
4. Data management: it collects and analyzes the data of different modules in different hospitals to realize the analysis and early warning of influenza in a systematic way. Moreover, it extracts various influenza corresponding data from the database, conducts in-depth exploration and calculation, and realizes the analysis and monitoring of the avian influenza epidemic.
5. Remote consultation management: it uses multimedia such as remote cameras to realize real-time remote consultation between hospitals at all levels and improve disease prevention and control. At the same time, it can also enable relevant decision makers to understand the epidemic information in a timely manner, strengthen the grasp of disease control information, and provide a reference for scientific decision-making. In summary, relevant decision makers can know the number of new flu patients, the number of people who have recovered, the status of disease changes, and the use of materials anytime and anywhere by querying the system in real time. In addition, relevant decision makers can also use various data analysis reports to calculate the utilization rate of hospital beds, the trend of medical supplies usage, and so on.

Through the flu real-time data collection and management system, we can get the number of infected and recovered people on each day of the cycle. These actual values often differ from the predicted values we made in the first stage. In order to more accurately portray the development trend of influenza, this section will use the collected real-time infection data to adjust the parameters of the prediction model to reflect the latest data on susceptible, infected, and recovered persons collected during the execution of the current cycle. There are four parameters in the SIRS model. *β* is the spread infection coefficient of an epidemic, which is generally determined through medical research. In particular, for unknown epidemic types, taking into account climate change and other factors, *β* will also change slightly over time. *γ* is the coefficient of recovery of infected persons. This parameter will gradually change as people's understanding of the flu epidemic increases and the cumulative number of recovered patients increases. *δ* is the coefficient of loss of immunity of the epidemic, and it will be updated continuously as the epidemic is gradually controlled. *λ* is the entry and exit rate of the population. The population enters *S*(*t*) at a rate of *λN* and exits at a rate of*λS*(*t*)+*I*(*t*)+*R*(*t*), so the total population of the area remains stable. This section will adjust the prediction model parameters *β*, *γ*, *δ*, *λ* in each cycle to update our prediction model to reflect the most recently observed data so that we can make the “best” prediction for the next cycle. In order to construct the parameter adjustment optimization model, we use the forecast results of the last day of the current cycle to construct constraints as follows:

(23) $$\begin{array}{c} \left\{\begin{array}{c} S\left(T\right)-\left[\begin{array}{c} S\left(T-1\right)+\lambda N-\beta S\left(T-1\right)\\ I\left(T-1\right)+\delta R\left(T-1\right)-\lambda S\left(T-1\right) \end{array}\right]=0,\\ I\left(T\right)-\left[\begin{array}{c} I\left(T-1\right)+\beta S\left(T-1\right)I\left(T-1\right)\\ -\gamma I\left(T-1\right)-\lambda I\left(T-1\right) \end{array}\right]=0,\\ R\left(T\right)-\left[\begin{array}{c} R\left(T-1\right)+\gamma I\left(T-1\right)-\\ \delta R\left(T-1\right)-\lambda R\left(T-1\right) \end{array}\right]=0. \end{array}\right) \end{array}$$

The above formula is a linear equation system of *β*, *γ*, *δ*, and *λ*. Among them, $\begin{array}{c} S\left(T\right),I\left(T\right),R\left(T\right),\\ S\left(T-1\right),I\left(T-1\right),R\left(T-1\right) \end{array}$ is the actual value that can be obtained, and the constraint condition can also be expressed as follows:

(24) $$\begin{array}{c} \left\{\begin{array}{c} S\left(T\right)-\hat{S}\left(T-1\right)\left(\beta ,\lambda ,\delta \right)=0,\\ I\left(T\right)-\hat{I}\left(T-1\right)\left(\beta ,\gamma ,\lambda \right)=0,\\ R\left(T\right)-\hat{R}\left(T-1\right)\left(\gamma ,\lambda ,\delta \right)=0. \end{array}\right) \end{array}$$

Here, the constraint indicates that the predicted number of people on the last day of the current planning cycle is equal to the actual number of people, that is, to ensure that the prediction error on the last day is zero. The objective function of the adjustment phase is to minimize the weighted forecast error of all days except the last day in the current period. The closer to the last day, the greater the weight assigned. The objective function is expressed as follows:

(25) $$\begin{array}{c} \min\sum_{t=1}^{T-1}w_{i}\left\{\begin{array}{c} {\left[S\left(T-t\right)-\hat{S}\left(T-t-1\right)\left(\beta ,\lambda ,\delta \right)\right]}^{2}+\\ {\left[I\left(T-t\right)-\hat{I}\left(T-t-1\right)\left(\beta ,\gamma ,\lambda \right)\right]}^{2}\\ +{\left[R\left(T-t\right)-\hat{R}\left(T-t-1\right)\left(\gamma ,\delta ,\lambda \right)\right]}^{2} \end{array}\right\}, \end{array}$$

(26) $$\begin{array}{c} \sum_{t=1}^{T-1}w_{t}=1,\;0<w_{T-1}<\ldots <w_{1}. \end{array}$$

The objective function is essentially a weighted moving average method, which can be used to reflect the most reliable basic forecasting principle of the latest data. In this section, the rank of the weight coefficient matrix is equal to the rank of the augmented matrix and is smaller than the number (*r*_*A*_=*r*_(*A|B*)_=2 < 4)of the constraint condition (24). This ensures the existence of the solution for constraint (25). The constraint condition (24) can produce a feasible region, which is the feasible solution set of the optimization subproblem. By solving the quadratic programming problems (24) (25), the optimal *β*^*∗*^, *γ*^*∗*^, *δ*^*∗*^, and *λ*^*∗*^ can be found for the next decision cycle, which can be used to accurately predict the next cycle.

So far, the FPEA model composed of forecasting, planning, execution, and adjustment stages has formed a cyclic system, which can be dynamically updated and planned and executed using the “dynamic decision-making framework.”

## 5. System Tests

This study takes a hospital as an example, and the data sources are all from that hospital. Moreover, this study uses 3 medical supplies, 1 hospital warehouse, 3 hospital departments, and 52 time points a year as the test background. The demand for the three kinds of medical materials all obeys the normal distribution. After running a Matlab program of a deterministic model, we can obtain the scheduling results of multiple medical supplies ordering and distribution based on random demand, as shown in Figure 4.

At the same time, we obtained the planning results for the ordering and distribution of three medical materials during the entire planning period (52 weeks), including the order quantity of the warehouse and each department's delivery quantity. In this section, we take item 1 as an example. As shown in Figure 5, the model systematically considers the constraints of the entire planning period to achieve a good balance between fixed order costs and inventory retention costs so as to obtain the minimum total operating cost of the hospital and the optimal ordering and distribution scheduling.

The planning results of multiple material stochastic models are shown in Figure 6. As the average value of demand continues to increase, the target value of the model also shows a rising trend. This phenomenon is the same as the two models of single determinism and single stochastic. It shows that when the demand increases, in order to reduce the impact of random disturbances, the hospital must order more medical supplies and increase more inventory, which leads to an increase in overall operating costs.

Under the condition of keeping the average value unchanged, the standard deviation sensitivity analysis of the demand is conducted, and the planning result is shown in Figure 7. The increase in the standard deviation rate of change represents an increase in random disturbances. In the process of increasing the standard deviation change rate from 80% to 120%, the target value of the random programming shows a rising phenomenon. Moreover, we can observe that the increase of the target value is constantly increasing. That is, when the standard deviation increases by a factor, the total operating cost will increase by a larger factor. Therefore, in actual operations, the greater the disruption to the demand for medical supplies, the more operating costs medical institutions will pay. This result also prompts medical institutions to minimize the interference of random factors on demand for medical supplies to ensure the overall stable operation of medical institutions.

The planning results of multiple material stochastic models are shown in Figure 8. In the process of increasing the fixed order cost from 80% to 120%, the target value gradually decreases, reaches the minimum at the rate of change equal to 90%, and then continues to rise. The reason for this phenomenon is the same as the single material random programming model, that is, when the fixed order cost increases, the hospital will reduce the order frequency in order to reduce the order cost, but each order quantity will increase, which causes the inventory cost to increase.

The planning results of multiple material randomness models are shown in Figure 9. As the average demand continues to increase, the target value of the model also shows a rising trend. This phenomenon, like the single determinism and single randomness models, shows that when demand increases, in order to reduce the impact of random disturbances, hospitals must order more medical supplies and increase inventory, which leads to an increase in overall operating costs.

Next, the performance of the model is verified, and the data processing speed is studied based on the high-frequency demand for medical supplies through 60 sets of data. There are more than 500 requirements in each set of data. First, we check the system's data processing speed, and the results are shown in Table 4 and Figure 10.

Figure 10 shows that the model constructed in this paper can basically meet actual needs in terms of data processing speed. Next, we perform statistics on the distortion rate of the data, and the results are shown in Table 5.

It can be seen from the data distortion rate statistics chart shown in Figure 11 that the data distortion rate of the model in this paper is below 0.05% during data processing, so the data transmission fidelity rate is high. Therefore, it can be seen that the system constructed in this paper has a certain application value.

## 6. Conclusion

In this study, a special system for artificial intelligence robot logistics is constructed. The space-time network structure is used to describe the medical supplies ordering and distribution logistics, and a deterministic O-1 mixed integer programming model of single varieties of materials is constructed. Because the model has the complex nature of NP-hard, this paper designs a heuristic algorithm to solve it effectively. Based on the deterministic model, this study introduces random medical supplies demand and considers the ordering and distribution of multiple varieties of supplies. Moreover, in order to better conform to the actual operating conditions of the hospital, this study uses the chance-constrained planning method to construct a random variety planning model of single-species and multispecies medical supplies. In the model solution, this paper uses the classic intelligent algorithm-genetic algorithm and executes the programming solution in the Matlab environment, which greatly improves the solution efficiency. Through the example test and sensitivity analysis of the three planning models, it can be concluded that the medical material ordering and distribution scheduling model constructed in this paper can effectively consider the random characteristics of medical material demand in actual operation and obtain effective medical material ordering and distribution operation results.

## Figures and Tables

**Figure 1:** Algorithm calculation process.

**Figure 2:** System technical architecture diagram.

**Figure 3:** System function module diagram.

**Figure 4:** The results of multiple materials stochastic model running once.

**Figure 5:** Ordering and distribution scheduling of the first medical supplies.

**Figure 6:** Demand average sensitivity analysis-multiple materials stochastic model.

**Figure 7:** Demand standard deviation sensitivity analysis-multiple materials stochastic model.

**Figure 8:** Sensitivity analysis of fixed order costs-multiple materials stochastic model.

**Figure 9:** Sensitivity analysis of demand average value-randomness model of multiple materials.

**Figure 10:** Statistical diagram of model data processing speed.

**Figure 11:** Statistical diagram of data distortion rate.

**Table 1:** Summary of modeling parameters.

*AM*, *NM*	The set of all nodes and nodes in the space-time network
*SW*	The collection of all nodes between the supplier and the hospital warehouse
*WD*	The collection of all nodes between the hospital warehouse and the department
*HA*	The collection of all stranded node lines
*p*	The unit purchase price of medical supplies
*d*	The unit distribution cost from warehouse to department
*h*_*w*_/*h*_*d*_	The unit inventory cost of medical materials in the warehouse/department
*c*	Fixed costs incurred for each order
*l*_*ij*_, *u*_*ij*_	The lower limit and upper limit of the flow of the node line (*i*, *j*)
*a*_*j*_	The demand amount of the *i*-th node
*x*_*ij*_	Flow of node line(*i*, *j*)
*δ*_*ij*_	0–1 variable indicating whether the hospital orders from the supplier

**Table 2:** Summary of modeling parameters.

*t*	The unit out-of-stock cost
*l*_*ij*_, *u*_*ij*_	The lower limit and upper limit of the flow of the node line (*i*, *j*)
*a*_*i*_	The demand amount at point *i*
*α*, *β*, *λ*	The confidence level of the corresponding opportunity constraint
*x*_*ij*_	The flow of the node line (*i*, *j*)
*y*_*i*_	The out-of-stock quantity at node *i*, $y_{i}=\max\left(a_{i}-\sum_{j\in WD}x_{ij},0\right),\;i\in D$
*δ*_*ij*_	0–1 variable indicating whether the hospital orders from the supplier

**Table 3:** Summary of second modeling parameters.

*AM* ^*n*^, *NM*^*n*^	The collection of all nodes and node lines in the nth layer of space-time network
*SW* ^*n*^	The collection of all node lines between the supplier and the hospital warehouse in the nth layer of space-time network
*WD* ^*n*^	The collection of all node lines between the hospital warehouse and departments in the nth layer of space-time network
*HA* ^*n*^	The collection of all stranded node lines in the nth layer of space-time network
*RM* ^*n*^	The unit purchase price of medical materials in the nth layer of space-time network
*D* ^*n*^	The unit distribution cost from warehouse to department in the nth time-space network
*n*, *N*	The set of the nth layer of spatiotemporal networks and the set of all spatiotemporal networks
*p* ^*n*^	The nit purchase price of medical materials in the nth layer of space-time network
*d* ^*n*^	The unit distribution cost from warehouse to department in the nth time-space network
*h*_*w*_/*h*_*d*_	The unit inventory cost of the medical materials in the warehouse/department in the nth time-space network
*c* ^*n*^	The fixed cost incurred for each order in the nth layer of space-time network
*t* ^*n*^	The unit out-of-stock cost in the nth time-space network
*um*_*ij*_	The maximum storage capacity of the hospital warehouse and department for the stranded node line (*i*, *j*)
*l*_*ij*_^*n*^, *u*_*ij*_^*n*^	The lower limit and upper limit of the traffic of the node (*i*, *j*) in the nth space-time network
*a*_*j*_^*n*^	The demand of the *i*-th node in the nth time-space network
*α*, *β*, *λ*	The confidence level of the corresponding opportunity constraint
*x*_*ij*_^*n*^	The flow of node line (*i*, *j*) in the nth layer of space-time network
*y*_*i*_^*n*^	The out-of-stock quantity of the *i*-th node in the nth time-space network
*δ*_*ij*_^*n*^	0–1 variable indicating whether the hospital orders from the supplier

**Table 4:** Model data processing speed.

No.	Data processing speed (ms)
1	95.5
2	77.2
3	98.9
4	94.6
5	83.2
6	95.5
7	73.4
8	90.0
9	78.3
10	91.7
11	93.0
12	96.8
13	78.9
14	82.6
15	75.1
16	91.7
17	66.8
18	87.8
19	68.7
20	74.3
21	91.9
22	96.8
23	87.0
24	85.6
25	84.5
26	80.4
27	76.0
28	73.2
29	78.1
30	75.3
31	73.9
32	67.5
33	68.0
34	84.5
35	96.7
36	84.7
37	84.1
38	68.6
39	91.5
40	65.1
41	66.3
42	81.6
43	68.6
44	94.2
45	75.4
46	97.3
47	66.7
48	91.1
49	66.2
50	84.0
51	89.2
52	68.9
53	97.0
54	94.2
55	76.1
56	97.0
57	82.9
58	88.6
59	83.0
60	75.4

**Table 5:** Statistical table of data distortion rate.

No.	Distortion (%)
1	0.004
2	0.044
3	0.016
4	0.043
5	0.018
6	0.042
7	0.003
8	0.009
9	0.048
10	0.033
11	0.015
12	0.021
13	0.002
14	0.022
15	0.016
16	0.001
17	0.023
18	0.029
19	0.025
20	0.006
21	0.023
22	0.006
23	0.028
24	0.025
25	0.013
26	0.005
27	0.040
28	0.028
29	0.027
30	0.049
31	0.028
32	0.024
33	0.000
34	0.038
35	0.047
36	0.010
37	0.031
38	0.011
39	0.017
40	0.020
41	0.037
42	0.021
43	0.005
44	0.041
45	0.029
46	0.004
47	0.039
48	0.028
49	0.002
50	0.007
51	0.015
52	0.047
53	0.045
54	0.043
55	0.028
56	0.008
57	0.050
58	0.002
59	0.004
60	0.044

## Data Availability

The authors were not given permission to share the data.
